# Efficacy, safety, and cost of surgical versus nonsurgical treatment for carpal tunnel syndrome: A systematic review and meta-analysis

**DOI:** 10.1097/MD.0000000000004857

**Published:** 2016-10-07

**Authors:** Yi-Ming Ren, Xi-Shan Wang, Zhi-Jian Wei, Bao-You Fan, Wei Lin, Xian-Hu Zhou, Shi-Qing Feng

**Affiliations:** a Department of Orthopedics, Tianjin Medical University General Hospital, Tianjin, China; b Department of Orthopedics, People's Hospital of Rizhao, Shandong, China.

**Keywords:** carpal tunnel syndrome, conservative treatment, meta-analysis, surgical release, systematic review

## Abstract

**Background:**

Carpal tunnel syndrome (CTS) is a common peripheral nerve entrapment disease. Either surgical or conservative intervention for CTS patients is needed to choose. We conducted this systematic review and meta-analysis to compare the clinical efficacy, safety, and cost of surgical versus nonsurgical intervention.

**Methods:**

The eligible studies were acquired from PubMed, Medline, Embase, Web of Science, Google, and Cochrane Library. The data were extracted by 2 of the coauthors independently and were analyzed by RevMan5.3. Standardized mean differences (SMDs), odds ratios (ORs), and 95% confidence intervals (CIs) were calculated. Cochrane Collaboration Risk of Bias Tool and Newcastle–Ottawa Scale were used to assess risk of bias.

**Results:**

Thirteen studies including 9 randomized controlled trials (RCTs) and 4 observational studies were assessed. The methodological quality of the trials ranged from moderate to high. The difference of clinical efficacy was statistically significant between surgical and nonsurgical intervention, and nonsurgical treatment was more effective (OR = 2.35, 95%CI = 1.18–4.67, *P* = 0.01). Meanwhile, different results were discovered by subgroup analysis. The pooled results of function improvement, symptom improvement, neurophysiological parameters improvement, and cost of care at different follow-up times showed that the differences were not statistically significant between the 2 interventions. The difference of complications and side-effects was statistically significant and conservative treatment achieved better result than surgery (OR = 2.03, 95%CI = 1.28–3.22, *P* = 0.003). Sensitivity analysis proved the stability of the pooled results.

**Conclusion:**

Both surgical and conservative interventions had benefits in CTS. Nonsurgical treatment was more effective and safety than surgical treatment, but there were no significant differences in function improvement, symptom improvement, neurophysiological parameters improvement, and cost of care. Nonsurgical treatment is recommended as the optical choice for CTS. If conservative treatment fails, surgical release can be taken.

## Abstract 2

Supplemental Digital Content is available in the text

## 1 Introduction

Carpal tunnel syndrome (CTS) is a pathological condition, caused by median nerve compression in the carpal tunnel at the wrist. As the most common peripheral nerve entrapment syndrome, CTS often occurs in middle-aged women with a female to male ratio of 2.07. Meanwhile, many jobs require workers to use vibrating tools or a firm grip, which may result in CTS.^[1–3]^ Although the incidence of this disease varied from 0.125% to 1% in the USA, recently, it has continued to increase annually.^[4]^ The most common symptoms include tingling, numbness, and pain within the 3 to 4 radial side fingers where median nerve distributed. When it becomes aggravating, weakness and atrophy of thinner muscles can occur, along with sensory loss in the affected fingers.^[5]^ There are no universally accepted diagnostic clinical and laboratory criteria so far, and diagnosis mainly relies on clinical symptoms and electro-diagnostic tests. In addition, CTS is not only caused by occupational tasks, but also associated with some systemic conditions, such as rheumatoid arthritis, hypothyroidism, diabetes, and pregnancy.^[6]^

The treatment of CTS consists of surgical release and nonsurgical treatment. The CTS patients, especially mild to moderate CTS patients, could choose surgical or conservative intervention. Usually, the patients with mild symptoms, short duration, and who not allowed to undergo surgery or not willing to accept the hand operation would choose conservative interventions, such as splinting, steroids, activity modification, nonsteroidal antiinflammatory drugs, diuretics, vitamin B6, ultrasound, and others.^[2]^ Nevertheless, only splinting and steroids approaches are supported according to high quality evidence.^[7,8]^ Surgical treatment is proven to be effective for patients with invalid conservative treatment or moderate to severe symptoms.^[9]^ However, sometimes patients worry about discomfort, inconvenience, or risks associated with surgical release, thus, they would rather choose conservative management.

In 2008 and 2011, Verdugo et al^[8]^ and Shi and MacDermid^[10]^ respectively published a systematic review based on relevant randomized controlled trials (RCTs) comparing the efficacy of surgical and nonsurgical treatment for CTS in improving clinical outcomes. To provide more evidence for clinical decision and an updated study, we conducted this systematic review and meta-analysis with more RCTs and related observational studies to compare the efficacy, safety, and cost of surgical versus nonsurgical intervention.

## 2 Materials and methods

Ethical approval or patient consent was not required since the present study was a review of previous published literatures.

### 2.1 Inclusive criteria of published studies

#### 2.1.1 Types of studies

We considered all published and unpublished studies covering RCTs, and observational studies including retrospective and prospective studies.

#### 2.1.2 Types of participants

All patients had been diagnosed as CTS, regardless of the diagnostic criteria used, etiology of the syndrome, associated pathology, gender, and age.

#### 2.1.3 Types of interventions

All surgical techniques including open carpal tunnel release (OCTR), endoscopic carpal tunnel release, and mini incision technique were considered. The nonsurgical treatment included: drugs – local steroid injection, vitamin B, diuretics, nonsteroidal antiinflammatory drugs, and others; laser therapy; wrist splinting; ultrasound therapy; and work modification/activity restriction, a hand therapist, exercises, a self-care booklet, and others. The studies comparing 2 surgical interventions or 2 nonsurgical managements, as well as those not providing sufficient data, were excluded.

#### 2.1.4 Types of outcome measures

The primary outcome measure was the clinical efficacy synthesizing clinical improvement, success rate, patients’ satisfaction, function, and symptom improvement (visual analogue scale [VAS] score, Carpal Tunnel Syndrome Assessment Questionnaire [CTSAQ]) at the last follow-up.

The secondary outcomes included: function and symptom improvement (symptom severity score, functional status score, and CTSAQ functional score); neurophysiological parameters improvement (median motor latency, median motor velocity, median sensory latency, and median sensory velocity); cost of care comparison; and complications and side-effects.

### 2.2 Search methods for the identification of studies

Six databases (PubMed, Medline, Embase, Web of Science, Google, and Cochrane Library) were searched using the keywords such as “carpal tunnel syndrome or Carpal tunnel syndrome,” “nerve entrapment or nerve compression,” “corticosteroid or steroid or injection,” “splint or splints or splinting,” “surgery or surgical or operation,” and “non-surgical or conservative” through July 2016 to collect relevant studies about the clinical comparisons of surgical versus nonsurgical intervention in CTS. Only English language papers were considered. The titles and abstracts of potential related articles identified by the electronic search were reviewed. References from retrieved articles were also assessed to extend the search strategy.

### 2.3 Data collection and quality assessment

Two partners (WL, BYF) independently assessed the titles and abstracts of all the studies screened during initial search, and they excluded any clearly irrelevant studies using the inclusion criteria. Data were independently extracted using a standard data form for the first author name, year of publication, sample size, gender, age, intervention, country, study design, follow-up, and relevant outcome. A 3rd partner (ZJW) would handle any disagreement about inclusion of a study and reach a consensus. Cochrane Collaboration Risk of Bias Tool^[11]^ was manipulated for the appraisal of RCT study quality. Observational studies were assessed by the Newcastle–Ottawa Scale including 8 items.^[12]^ A higher overall score indicates a lower risk of bias and a score of 5 or less (out of 9) corresponds to a high risk of bias.

### 2.4 Statistical analysis

RevMan statistical software5.3 was used for meta-analysis. The continuous variables would be conducted by standardized mean differences (SMDs) and 95% confidence intervals (CIs). For the dichotomous outcome, we calculated the odds ratios (ORs) and 95% CIs. We selected SMD not weighted mean difference causing that these included studies used different measurement indexes for efficacy assessment. The Chi-squared statistic and the *I*^2^ statistic were used for the test of heterogeneity. A *P* < 0.05, *I*^2^ > 50% was considered a significant heterogeneity, and random-effect models were applied. Otherwise fixed-effect models were used if there was no significant heterogeneity (*P* ≥ 0.05, *I*^2^ ≤ 50%). Subgroup analyses based on study of type, duration of follow-up, and nonsurgical interventions were performed comparing RCT to retrospective study, follow-up duration ≤12 to >12 months, and different nonsurgical interventions. We also performed sensitivity analysis to assess the stability of the results and investigate the influence of each study by omitting a single study sequentially. Publication bias was showed by funnel plot.

## 3 Results

### 3.1 Studies identification and inclusion

Searches conducted in the PubMed, Medline, Embase, Web of Science, Google, Cochrane Library databases, and other sources yielded a total of 2411 articles. After removing duplicates, 746 literatures were remained. Based on the titles and abstracts review, 722 irrelevant articles and 2 systematic reviews of them were excluded. Twenty-two full-text articles were assessed for eligibility. However, 9 articles were excluded based on the previously established exclusion criteria (5 without available data, 4 without comparison between surgical and nonsurgical treatment). Finally, 13 trials (9 RCTs and 4 observational studies) were included in this systematic review and meta-analysis. The detail of selection process is listed in Fig. 1.

**Figure 1:** Preferred Reporting Items for Systematic Reviews and Meta-Analyses (PRISMA) flow diagram.

### 3.2 Study characteristics

We assessed 13 studies including 9 RCTs, 2 retrospective studies, and 2 comparative cohort studies in this article. Overall, 5 studies compared surgery with steroid injection, 4 studies about surgery versus multimodality, 3 studies about surgery versus splinting, and 1 study about surgery versus laser therapy. The included studies were conducted in 8 countries (Pakistan, Spain, USA, Egypt, Netherlands, Turkey, Hong Kong, and UK) from 1964 to 2015, and involved 1246 patients (542 patients treated with surgery, 704 patients treated with conservative intervention) aged 32.8 to 51.53 years. The average follow-up duration ranged from 1 to 54 months. The primary clinical outcomes were not consistent among the identified studies, so we synthesized function and symptom improvement (VAS score, CTSAQ) in Jarvik et al, Ly-Pen et al, and Awan et al articles,^[13–15]^ clinical improvement in Garland et al and Seradge articles,^[16,17]^ success rate in Gerritsen et al article^[18]^ and patients satisfaction in Halil et al article^[19]^ at the last follow-up to compare the clinical efficacy. For secondary outcomes, we pooled the data of function and symptom improvement (symptom severity score, functional status score, and CTSAQ functional score), neurophysiological parameters improvement, cost of care comparison, complications, and side-effects. The detailed information of included studies is shown in Table 1.

**Table 1:** Characteristics of studies included.

### 3.3 Methodological assessment of study quality

Methodological quality assessment of the 13 included studies is presented in Fig. 2 and Table 2. Among the RCTs, most studies clearly described the random sequence generation by random number tables, blinding, and allocation concealment by sealed opaque envelopes containing the treatment allocation. Only Awan et al and Garland et al articles^[15,16]^ showed unclear information about that. Among the observational studies, scores of all 4 studies on the Newcastle–Ottawa scale assessing risk of bias, ranged from 7 to 9, indicating a low risk of bias.

**Figure 2:** Risk of bias summary: this risk of bias tool incorporates the assessment of randomization (sequence generation and allocation concealment), blinding (participants and outcome assessors), incomplete outcome data, selective outcome reporting, and other risk of bias. The items were judged as “low risk,” “unclear risk,” or “high risk.” Green means “low risk,” red means “high risk,” and yellow means “unclear risk.”

**Table 2:** Risk of Bias Assessment of Observational Studies.

### 3.4 Primary outcome: clinical efficacy

The clinical efficacy measures differed in the 7 included studies.^[13–15,16–19]^ Ly-Pen et al^[14]^ and Awan et al^[15]^ used the VAS rating system, and increases over 20% were related with symptom improvement. Jarvik et al^[13]^ used the 9-item functional status scale of the CTSAQ, and this scale is reliable and responsive to clinical change. In addition, patient amounts of clinical improvement in Garland et al and Seradge articles,^[16,17]^ success rates of patients treated in Gerritsen et al article^[18]^ and patients’ satisfaction percentages in Halil et al article^[19]^ were all included to compare the clinical efficacy. In Fig. 3, 7 included studies consisting of 782 CTS patients (336 patients received surgery and 446 patients received conservative treatment) investigated the clinical efficacy at the last follow-up. A significant heterogeneity among studies (*P* = 0.0009, *I*^2^ = 74%) was found, so we used the random effect model to pool the data. The overall estimate indicated that the pooled OR was 2.35 (95%CI = 1.18–4.67, *P* = 0.01), suggesting that the difference between the 2 groups was statistically significant, and nonsurgical treatment is more effective than surgical treatment.

**Figure 3:** Forest plot of comparison: clinical efficacy between surgery group and nonsurgery group.

### 3.5 Primary outcome: subgroup analysis

We conducted 4 subgroup analyses for the clinical efficacy by type of study (RCT vs retrospective study), duration of follow-up (≤12 months vs >12 months), different nonsurgical interventions, and different continents. In the subgroup analyses by study of type (RCT: OR = 2.58, 95%CI = 1.04–6.41, *P* = 0.04; retrospective study: since only 1 study included, results are no need to show) (Fig. 4) and duration of follow-up (≤12 months: OR = 3.61, 95%CI = 0.74–17.52, *P* = 0.11; >12 months: OR = 1.94, 95%CI = 1.30–2.91, *P* = 0.001) (Fig. 5), the pooled results by type of RCTs and follow-up duration >12 months were in accordance with the overall estimate. However, the pooled results of the clinical efficacy of follow-up duration ≤12 months showed that there was no significantly statistical difference between patients treated with surgery and patients treated with conservative treatment. The heterogeneity of follow-up duration >12 months significantly decreased (*P* = 0.36, *I*^2^ = 1%), suggesting that the short follow-up time was the source of heterogeneity. The subgroup analysis by different nonsurgical interventions included 3 comparisons (surgery vs steroid injection; surgery vs splinting; and surgery vs multimodality) in Fig. 6. The subgroup analysis results of surgery versus splinting (OR = 4.88, 95%CI = 1.43–16.65, *P* = 0.01) and surgery versus multimodality (OR = 3.15, 95%CI = 1.23–8.07, *P* = 0.02) were also in accordance with the overall estimate. But the subgroup analysis result of surgery versus steroid injection (OR = 0.85, 95%CI = 0.41–1.77, *P* = 0.67) suggested that the difference between the 2 groups was not statistically significant. The heterogeneity of surgery versus steroid injection (*P* = 0.19, *I*^2^ = 43%) and surgery versus splinting (*P* = 0.14, *I*^2^ = 49%) decreased, suggesting that the comparison of surgery versus multimodality was the source of heterogeneity. A subgroup analysis of different continents in Fig. 7, containing USA versus Europe (Spain, Nederland, and UK) versus Pakistan. The subgroup analysis results of USA (OR = 3.15, 95%CI = 1.23–8.07, *P* = 0.02) and Europe (OR = 3.08, 95%CI = 1.12–8.46, *P* = 0.03) were also in accordance with the overall estimate. But the subgroup analysis result of Pakistan (OR = 2.35, 95%CI = 1.18–4.67, *P* = 0.18) suggested that the difference between the 2 groups was not statistically significant.

**Figure 4:** Forest plot of comparison: subgroup results of clinical efficacy by type of randomized controlled trials (RCTs) between surgery group and nonsurgery group.

**Figure 5:** Forest plot of comparison: subgroup results of clinical efficacy by duration of follow-up (≤12 vs >12 months) between surgery group and nonsurgery group.

**Figure 6:** Forest plot of comparison: subgroup results of clinical efficacy by different nonsurgical interventions (steroid injection vs splinting vs multimodality) between surgery group and nonsurgery group.

**Figure 7:** Forest plot of comparison: subgroup results of clinical efficacy by different continents containing USA versus Europe versus Pakistan between surgery group and nonsurgery group.

### 3.6 Secondary outcome: function and symptom improvement

Four included studies^[13,18,19,25]^ including 182 surgery group cases and 207 nonsurgery group cases provided the data in terms of symptom improvement in 6 months. A heterogeneity test revealed that a significant heterogeneity existed among the studies (*P* < 0.00001, *I*^2^ = 89%) and the random-effect model was used. A pooled analysis revealed that there was no significant difference between surgery and nonsurgery group (SMD = −0.35, 95%CI = −1.01–0.31, *P* = 0.30) (Fig. 8A). Comparison of functional improvement in 6 months between the 2 groups was conducted among 5 included studies,^[13,18,19,24,25]^ which contain 493 patients (212 patients received surgery and 281 patients received nonsurgery treatment) in Fig. 8B. A significant heterogeneity was found among studies (*P* < 0.00001, *I*^2^ = 91%), so the random-effect model was used. The pooled result showed that the difference between surgery and nonsurgery group was not statistically significant (SMD = −0.10, 95% CI = −0.73–0.52, *P* = 0.75).

**Figure 8:** (A) Forest plot of comparison: symptom improvement in 6 months between surgery group and nonsurgery group. (B) Forest plot of comparison: functional improvement in 6 months between surgery group and nonsurgery group. (C) Forest plot of comparison: improvement of median sensory latency between surgery group and nonsurgery group. (D) Forest plot of comparison: improvement of median sensory velocity between surgery group and nonsurgery group. (E) Forest plot of comparison: improvement of median motor latency between surgery group and nonsurgery group. (F) Forest plot of comparison: improvement of median motor velocity between surgery group and nonsurgery group. (G) Forest plot of comparison: cost of care between surgery group and nonsurgery group.

We also compared symptom improvement and functional improvement in 3 and 12 months, the overall estimates showed that the differences between the 2 groups were not statistically significant in Figures S1–S4 (presented as Supplementary files).

### 3.7 Secondary outcome: neurophysiological parameters improvement

Median sensory latency improvement was reported in 2 studies^[18,25]^ containing 205 patients. There was no significant difference in median sensory latency improvement between the 2 groups (SMD = −0.19, 95%CI = −1.21–0.84, *P* = 0.72) in Fig. 8C. A significant heterogeneity was found among the studies (*P* = 0.0003, *I*^2^ = 92%), so we used the random-effect models.

In Fig. 8D, 3 included studies^[19,23,25]^ consisting of 174 patients (92 patients received surgery and 82 patients received conservative treatment) investigated median sensory velocity improvement. A significant heterogeneity among studies (*P* = 0.02, *I*^2^ = 75%) was found, so we used the random-effect model to pool the data. The overall estimate indicated that the pooled SMD was 0.36 (95%CI = −0.29–1.00, *P* = 0.28), suggesting that conservative treatment and surgery had no statistically significant difference.

Comparison of median motor latency improvement between surgery and conservative treatment was conducted among 4 included studies^[18,19,23,25]^ which contain 307 patients in Fig. 8E. A heterogeneity test showed that there was the moderate heterogeneity among studies (*P* = 0.16, *I*^2^ = 41%), so the fixed-effect model was used. The overall estimate showed that the difference between the 2 groups was not statistically significant (SMD = −0.01, 95%CI = −0.23–0.22, *P* = 0.96).

Median motor velocity improvement was reported in 2 studies^[19,25]^ consisting of 124 patients in Fig. 8F. There was no significant difference in median motor velocity improvement between the 2 groups (SMD = −0.01, 95%CI = −0.59–0.57, *P* = 0.97). A moderate heterogeneity was found among the studies (*P* = 0.15, *I*^2^ = 51%), so we used the random-effect models.

We also compared median sensory velocity, median motor latency, and median motor velocity improvement in 3 months, the overall estimates showed that the differences between surgery and nonsurgery group were not statistically significant in Figures S5–S7 (presented as supplementary files).

### 3.8 Secondary outcome: cost of care comparison

Comparison of cost of care between surgery and conservative treatment was conducted among 2 included studies^[20,22]^ which contain 287 patients (139 patients received surgery and 148 patients received conservative treatment) in Fig. 8G. The heterogeneity test showed that there was no heterogeneity among studies (*P* = 0.74, *I*^2^ = 0%), so the fixed-effect model was used. The overall estimate showed that the difference between the 2 groups was not statistically significant (SMD = −0.12, 95%CI = −0.35–0.12, *P* = 0.33).

### 3.9 Secondary outcome: complications and side-effects

In Fig. 9, 7 included studies^[13,14,17–19,21,23]^ consisting of 864 CTS patients (367 patients received surgery and 497 patients received conservative treatment) reported complications or side-effects. A low heterogeneity among studies (*P* = 0.33, *I*^2^ = 13%) was found, so we used the fixed-effect model. The overall estimate indicated that the pooled OR was 2.03 (95% CI = 1.28–3.22, *P* = 0.003), suggesting that the difference was statistically significant, and the safety of nonsurgical intervention was better than that of surgery.

**Figure 9:** Forest plot of comparison: complications and side-effects between surgery group and nonsurgery group.

### 3.10 Sensitivity analysis and publication bias

We performed a sensitivity analysis to assess the stability of the pooled results. Among the most studies, the heterogeneity results were not obviously altered after sequentially omitting each study. In the pooled results comparing median sensory velocity improvement in 6 months, the heterogeneity significantly decreased (SMD = 0.70, 95%CI = 0.33–1.07, *P* = 0.56, *I*^2^ = 0%) after excluding the Hui study.^[23]^ So, Hui article was regarded as the source of heterogeneity. Similarly, Gerritsen et al study^[18]^ was considered as the source of heterogeneity because the heterogeneity significantly decreased after excluding it in the pooled results comparing symptom improvement in 6 months (SMD = −0.59, 95% CI = −0.86–0.32, *P* = 0.43, *I*^2^ = 0%). The funnel plot of the included studies^[13–19]^ is shown in Fig. 10. The points in the funnel plot were symmetrically distributed, indicating that the publication bias was not apparent.

**Figure 10:** Funnel plot to test for publication bias. Each point represents a separate study for the indicated association. Log OR represents the natural logarithm of the OR. The vertical line represents the mean effects size. OR = odds ratio, SE = standard error.

## 4 Discussion

### 4.1 Summary of main results

In this study, we identified 9 RCTs and 4 observational studies for investigating the efficacy, safety, and cost of surgical versus nonsurgical intervention. Our meta-analysis results showed that in RCTs or follow-up duration >12 months or surgery versus splinting and surgery versus multimodality, there was a significant difference between the 2 groups in the primary outcome, and the nonsurgery group proved it had a higher efficacy. However, different results were discovered by subgroup analysis. The subgroup result of follow-up duration ≤12 months showed that surgical versus nonsurgical intervention were equally effective, which may be caused by the shorter follow-up time. The subgroup result of surgery versus steroid injection indicated that the treatment effect of steroid injection approached to surgery, which demonstrated that steroid injection treatment may be better than other nonsurgical treatment. In addition, the subgroup results of different continents showed that nonsurgical intervention was better in USA and Europe, but surgical versus nonsurgical intervention were equally effective in Pakistan.

For secondary outcomes, the comparisons of surgical versus nonsurgical intervention in function improvement, symptom improvement, neurophysiological parameters improvement, and cost of care at different follow-up times resulted in the same performance. However, Pomerance and Zurakowski^[20]^ retrospectively compared direct costs for CTS patients with surgery versus nonsurgical care. The economic evaluation was performed from a societal perspective and involved all relevant costs between surgery group and splint group in Gerritsen and coworkers study.^[22]^ Based on the cost–utility ratio, they all summarized that surgery was more cost-effective, and recommended as the preferred treatment for CTS patients.

Complications and side-effects in 7 included studies also should be discussed. The meta-analysis result of complications and side-effects showed that there was a significant difference between the 2 groups. In Ly-Pen et al study,^[14]^ 8 patients in each group at the 2-week visit reported local pain at the wrist, which were resolved spontaneously during the following few days. As for minor adverse effects in Hui study,^[23]^ in the injection group 1 patient developed cellulitis, which was resolved with antibiotic treatment, and 4 (16%) had pain at the injection site. In the surgical group, 2 patients had wound hematoma and 9 (36%) had mild to moderate wound pain at 1 week but this had been resolved by the end of 6 weeks. Fortunately in Elwakil et al study,^[21]^ they only reported the scar-related complications in surgery group. Three hands of patients (10%) were affected by the occasional scar tenderness, and only 1 hand of patients (3.33%) was affected by the scar hypersensitivity. In Halil et al study,^[19]^ 2 patients coming from OCTR group had some postoperative problems. The rare complex regional pain syndrome was reported in 1 patient, and it was diagnosed by 3-phase bone scintigraphy. In the 1st week postoperatively, the scar tenderness of the other patient was discovered, but spontaneous improvement of this pain was reported after a few weeks. In Gerritsen et al study,^[18]^ 53 patients in the surgery group experienced a painful or hypertrophic scar and 24 patients were attacked by stiffness of the wrist, hand, or fingers. In the splinting group, 31 patients had stiffness of the wrist, hand, or fingers. Although many patients reported adverse effects, most of these were relatively mild and lasted only a short duration. However, 1 patient in the surgery group developed reflex sympathetic dystrophy. In Jarvik et al and Seradge studies,^[13,17]^ there were no clinically important adverse events and no surgical complications reported in either group. In summary, the safety of nonsurgical intervention was better than that of surgery.

Surgical treatment including OCTR, endoscopic carpal tunnel release, and minimal invasive techniques can reduce pressure on median nerve by cutting the transverse carpal ligament to increase space in carpal tunnel. For the majority of patients, surgery leads to symptomatic improvement, relief, and better function. Fortunately, with the development of minimal invasive techniques, incision and complication rate decreased significantly. Padua et al^[26]^ confirmed that even without any treatment, symptoms of 21% CTS patients can still improve after resting about 10 to 15 months. This showed that mild CTS had a certain rate of self-healing just by resting. Angelis et al^[27]^ affirmed that symptoms, function, and median nerve sensory conduction velocity of CTS patients improved after splinting for 3 or 6 months. Therefore, the authors recommended wearing a splint for 3 months, without long-term wear. Piazzini et al^[28]^ showed that vitamin B6 had no effect on CTS patients. Chang et al^[29]^ reported that oral steroids were the most effective among oral medicine. However, the side effects of large doses and toxins from the steroids were serious, and it was necessary to find a low-dose and short-term treatment. Many reports supported that local steroid injection resulted in improvement for CTS patients. It was reported that the symptom remission rate of CTS patients after local steroid injection for 1 year was 84.4%. Nevertheless, such a high effective rate was temporary, as it tends to recur at any time.^[30]^ The thermal effect of laser therapy and ultrasound therapy can promote venous return and reduce the edema in the carpal tunnel,^[31]^ but there was no enough evidence to show if there was a good effect. We concluded that severe CTS can be cured by radical surgery, but conservative interventions with comparable efficacy indeed alleviated symptoms continuously.

### 4.2 Comparison with previous studies

To our knowledge, this is the first systematic review and meta-analysis with moderate or high quality RCTs and observational studies to compare the efficacy, safety, and cost of surgical versus nonsurgical intervention for CTS. A meta-analysis of 4 RCTs published in 2008 by Verdugo et al^[8]^ found that the pooled estimate of clinical improvement and neurophysiological parameters improvement favored surgery, and the incidence of complications were significantly more common in the surgical arm. Our study including more RCTs showed that surgical and nonsurgical treatment had the same performance for neurophysiological parameters improvement. Four included studies in Verdugo study^[8]^ only compared surgery versus local steroid injection or splinting. In our study, conservative interventions included not only local steroid injection and splinting, but also low level laser therapy and multimodality. Another previous meta-analysis published in 2011 by Shi et al^[10]^ included 5 RCTs and 2 controlled trials, and they compared the improvement of patient self-administered scales, electrophysiological studies, complication, and side effect between surgical and nonsurgical treatment without subgroup analysis, sensitivity analysis, and publication bias analysis. In meta-analyses, adding more information from observational studies may aid in clinical reasoning and establish a more solid foundation for causal inferences.^[32]^ Our study including more RCTs and observational studies made subgroup analysis based on study of type, duration of follow-up, and nonsurgical interventions for further assessment. We also performed sensitivity analysis to assess the stability of the results and funnel plot was made to reveal the publication bias.

### 4.3 Limitations of the study

Some limitations of this study should be noted. First, significant statistical heterogeneity of function improvement, symptom improvement, and neurophysiological parameters improvement still existed among the included trials, which may be explained by the clinical diversity among trials. Second, there were no universal standardized metrics to assess the clinical primary outcome in the included studies, which may influence the reliability of the results in this study. Third, our study ignored the diversity of used diagnostic criteria and etiology of the syndrome, and further research is needed to discover whether these conclusions apply to patients with varying degrees of symptoms or idiopathic CTS patients. Last but not least, for conservative treatment, published researches mainly focused on the local steroid injection and splinting. Having less research about surgery versus other conservative interventions has limited this study's comprehensiveness.

## 5 Conclusions

In conclusion, this is the most comprehensive meta-analysis to date to show that nonsurgical treatment performed better efficacy and safety than surgical treatment, but no obvious differences were noted about function improvement, symptom improvement, neurophysiological parameters improvement, and cost of care. Nonsurgical treatment is recommended as the optical choice for CTS. If conservative treatment fails, surgical release can be taken. In view of the heterogeneity and different follow-up time, whether these conclusions are applicable should be further determined in future studies.

## Acknowledgments

The authors thank Program for Research Sponsored by the Health Authority of Binhai New Area of Tianjin, China (2012BWKY028), the State Program of National Natural Science Foundation of China (81371957), the State Key Program of the National Natural Science Foundation of China (81330042), the Special Program for Sino-Russian Joint Research Sponsored by the Ministry of Science and Technology, China (2014DFR31210), and the Key Program Sponsored by the Tianjin Science and Technology Committee, China (13RCGFSY19000, 14ZCZDSY00044) for the support.

## Supplementary Material

Supplemental Digital Content
